# Application of Personal Information Privacy Protection Based on Machine Learning Algorithm

**DOI:** 10.1155/2022/6710631

**Published:** 2022-07-31

**Authors:** Fang Lang, Yunfei Zhong

**Affiliations:** ^1^Law School of Weifang University, Weifang 261061, China; ^2^Shandong Weifang Tobacco Co Ltd., Weifang 261061, China

## Abstract

Based on a machine learning algorithm, this paper deeply explores the privacy protection of personal information. In this paper, the definition of the machine learning algorithm is put forward, the design idea of privacy protection in joint machine learning platform is studied, and the architecture model and model parameter updating strategy of joint machine learning under privacy protection are designed. To protect the privacy of personal information, this paper also proposes a data homomorphic verification mechanism to prevent the global parameters from being tampered with by malicious cloud servers. In order to verify the performance of the models constructed in this paper, the comparative experiments of different models are carried out. The experimental results show that this algorithm has a fast convergence speed, and the average error rate decreases by 4.17% compared with the traditional algorithm. Moreover, the accuracy of this algorithm reaches 95.37%, which is about 8.76% higher than the previous algorithm. This model is applied to the field of personal information privacy protection, which can provide a safe and reliable environment for personal information privacy and effectively protect the privacy of data owners. And, means and reference value is provided for the development direction of privacy protection.

## 1. Introduction

The amount of data generated by all walks of life is exploding as we enter the information age, thanks to the development of information technology such as the Internet; with the enhancement and aggravation of online data behavior, the protection of personal information and privacy is particularly prominent in the contemporary era [1]. As a result, the purposeful collection, investigation, utilization, transmission, disclosure, and sale of personal information via the Internet has reached an unprecedented level. Although easy-to-obtain personal data have become a staple of academia and industry, the process of data collection, publication, processing, and storage will be aided by a slew of third-party service providers, expanding the number of possible data sources [2]. Personal data collection, expansion, mining, and use for more precise business marketing activities have gradually become a new focus of business development for traditional businesses, Internet businesses, data-related businesses, and so on. With business's continued growth and prosperity, it also brings with it potential conflicts of interest and hidden risks for various individuals [3]. In addition, due to the prevalence of online fraud, user privacy breaches do occur from time to time. Personal privacy protection has become one of the problems brought on by the information society in the network environment. Despite the fact that the definition of privacy is complex and varied, personal information plays an important role in privacy [4]. The abuse and control of information is a major concern in today's world of privacy. People are gradually becoming more aware of personal privacy as big data-related technologies advance. As a result, countries' focus in formulating laws and regulations on privacy protection has shifted to how to properly protect privacy without impeding network development.

The content of privacy right is extensive, including the information secret of a natural person's personal life, the peace of his personal life, and even his own decision on private life. Therefore, from the content, the right to privacy can be said to be a collection of rights [5]. Personal information may be infringed in the commercial data behavior of Internet enterprises, that is, personal information risk; that is, personal information may be harmed as an Internet user. In the traditional differential privacy model, data from different sources are concentrated in the central server, and then the data are treated with privacy protection, and the central server publishes the inquiry information satisfying the differential privacy [6]. However, in the process of data collection, third-party service providers are often uncontrollable, which easily leads to privacy leakage [7]. The characteristics of diverse data sources, fragmented information, and personalized and differentiated privacy requirements lead to the risk of privacy leakage when multi-party data are merged. At the same time, the separation of data ownership and storage rights, multisource, high-dimensional, and dynamic characteristics aggravate the risk of privacy leakage in the process of data sharing and pose new challenges to privacy protection technology. Personal information, as an original part of “privacy,” has become a prominent contemporary problem in the background of the increasingly prosperous enterprise data behavior [8]. At the same time, data privacy has become the core issue of machine learning, especially when using some sensitive data in cloud computing, the cloud is not completely trustworthy. Therefore, privacy protection and machine learning algorithms must be designed for the cloud. Machine learning provides a potentially powerful framework for automated perception and reasoning. However, a good machine learning framework still needs a large number of data sets to fully realize its potential of perception and reasoning. In this paper, a personal information privacy protection model based on a machine learning algorithm is constructed, and its innovations are as follows:

① This paper studies the structure design and working mechanism of distributed machine learning system under privacy protection and analyzes the design strategy of privacy protection in a distributed machine learning system. Aiming at the privacy protection of personal information, this paper designs a data homomorphic verification mechanism to prevent the global parameters from being tampered by malicious cloud servers.
② This paper investigates vector addition, number multiplication, linear transformation, and weighted inner product homomorphism operations using vector homomorphism encryption; this allows the vector homomorphic encryption scheme to meet the basic operations in machine learning. A local differential privacy data stream protection protocol is proposed that can provide data stream privacy while also ensuring high data availability and requiring less storage and computing power.

This paper mainly explores the privacy protection of personal information, which is divided into five sections. The specific research framework is as follows:

Section 1 is the introduction. This part introduces the research background, significance, and methods of this paper and gives the innovation and organizational structure of this paper.  Section 2 is a summary and research of related literature at home and abroad and introduces the research methods of this paper.  Section 3 mainly constructs the privacy protection model of personal information based on a machine learning algorithm. Among them, Section 3.1 analyzes the concept connotation of privacy protection and machine learning and summarizes the related basic theories.  Section 3.2 focuses on the construction method and implementation of the personal information privacy protection model.  Section 4 is the experimental analysis. In this part, many experiments are carried out, and the experimental results of other models are compared to analyze the performance of the models.  Section 5 is the conclusion and prospect. This part mainly reviews the main contents and results of this research, summarizes the research conclusions, and points out the direction of further research.

## 2. Related Work

The arrival of the information age has brought about changes in all aspects of our lives, and profound business changes have taken place in the global society. With the rapid growth of intelligent terminal devices, massive data are generated anytime and anywhere. These data have profound value, and all kinds of enterprises and institutions begin to collect personal data on a large scale and analyze and mine the collected data. While enjoying the convenience brought by information technology, information security and privacy have become the focus of people's attention. Therefore, many researchers have made relevant explorations on data search and personal information privacy protection technology.

Ocansey et al. [9] proposed a fully dynamic fully homomorphic encryption scheme that no longer limits the number of allowable parties [9]. Wang et al. [10] propose an outsourced secure multi-party computation framework. The scheme uses two noncollusion cloud servers, one for storage and computing, and the other contains the master private key that can decrypt user data and realizes computing outsourcing by constructing a secure protocol [10]. Wang et al. [11] proposed a security outsourcing detection system, the system classification is completed by the support vector machine algorithm, and privacy protection is achieved by designing a secure multiparty protocol [11]. Yin et al. [12] focused on data outsourcing services on the basis of analyzing the risks of privacy leakage in the stages of data release, storage, and search and combined with the multiparty requirements for data privacy protection granularity, data availability, timeliness, and other dimensions at different stages. Research on key technologies of data privacy protection under the mode [12]. Reza et al. [13] took the hybrid cloud as the data bearing platform, proposed a data segmentation technology based on the k-anonymity criterion, and designed a complete set of data anonymity segmentation scheme to solve the balance of data privacy protection and availability when the set-valued data is released [13]. Wei et al. [14] believe that attackers can obtain data privacy by filtering random noise. Furthermore, random perturbations may expose the privacy of outliers when attackers have access to external information, i.e., published data about individuals may contain quasi-identifier properties that may be linked to public databases to reidentify individual records [14]. Liu and Zhou [15] proposed a privacy protection scheme based on differential privacy, and its protection of data privacy has nothing to do with the background knowledge mastered by the attacker. This scheme ensures that statistical queries on the target dataset and on datasets that differ by only one record are identical in results [15]. Ke et al. [16] proposed the use of differential privacy computing to achieve privacy-preserving mining of joint datasets [16]. Barni et al. [17] proposed a distributed algorithm, which assumes that the same record has a unique global identifier in a vertically divided data environment, and all parties involved in data fusion only have data with partial attributes; the original information is hidden in the communication process, and the privacy protection of the data fusion process is realized by constructing a complete anonymity table to determine whether the anonymity threshold is met [17]. Hu et al. [18] proposed an algorithm for users to learn game equilibrium. The classifier built by this algorithm enables each user to strike a balance between the accuracy of the classification task and data privacy [18]. Xie et al. [19] proposed an abstract model to support databases with any number of public and private variables and formulated application-independent privacy protection granularity and utility metrics, where privacy protection granularity was quantified by ambiguity, and data utility was measured by Fidelity to quantify [19].

Based on research on privacy protection of personal information in related literature studies, this paper proposes a new research approach and method. Using the machine learning architecture model, this paper creates the overall architecture of the joint machine learning platform, as well as the key structure of the central server. A fast synchronous random gradient descent method is designed for a heterogeneous multiclient situation to ensure fast training and convergence of the model, as well as to improve the generalization ability of the existing model. The traditional disturbance mechanism is used to protect the key attribute data, with noise satisfying the definition of local differential privacy added to the model's local update. As a result, the aggregation operation can be used to initialize the global model parameters, resulting in fewer model training communication rounds. Experiments show that the model is stable and reliable, as well as that it performs as expected.

## 3. Methodology

### 3.1. Privacy Protection and Machine Learning

As a contributor of individual knowledge and content, participate in knowledge creation and sharing in the information age. At the same time, with the help of the Internet, individuals can realize some or all activities or projections in reality and conduct business transactions, self-construction, social interaction, information acquisition, and other actions. At present, the collection, expansion, mining, and use of personal information for more accurate business marketing activities has gradually become a new focus of business development for traditional enterprises, Internet companies, data-related enterprises, and so on [20]. With the continuous development and prosperity of business, it also brings potential conflicts of interests and risks of different individuals. Internet privacy refers to the right that a natural person enjoys on the Internet that his personal affairs are not publicly publicized, his private life is not disturbed, and his personal information related to online activities is protected from being illegally collected, known, utilized, and disclosed by others. In the information age, massive data have brought obvious privacy security problems in the practical application of machine learning. Users' personal highly sensitive data are collected and kept in commercial companies indefinitely. Users can neither delete these data nor restrict the use of them by commercial companies. Considering the privacy and security of data, many data holders are reluctant to share their data sets, so they can not directly use the joint data sets of participants for machine learning [21]. As an important component of the original concept of privacy, personal information will face more prominent and severe challenges in the information age and networking. The new emphasis of network privacy in the era lies in the problem of “privacy digitalization” brought by network society. This is the core issue of “privacy” in the information age.

In the information age, the right of network privacy should include the following aspects: ① the control of personal information. ② The right to be free from interference when individuals conduct online behavior. ③ The obligee's knowledge of the use and collection of personal information on the Internet by others, and his request to withdraw from deletion, etc. In the network society, the mass production of personal information and the precipitation of structured and unstructured data make it possible to use data to analyze consumer behavior and preferences and increasingly move towards accurate consumer description and database marketing. The more accurate you understand the marketing audience, the more you can achieve the marketing management goal of low cost and high return. With the development of cloud computing technology, it has gradually become a trend for enterprises to go to the cloud [22]. Personal information such as users' personal photos, home address, contact information, etc., may be permanently stored in the company server of the cloud service provider, which is beyond the control of the owner. The violations of users' privacy rights involved in the management of network resources mainly include improper use of network users' personal information, privacy of personal activities, traces of personal networks, and infringement of personal cyberspace. The collected person of personal information has the right to ask the collector to take necessary and reasonable measures to protect the security of his personal data. First of all, you can ask the website to take certain technical measures and policies to keep the collected data; secondly, their personal data shall not be transmitted or disclosed to any third party; finally, within the network service group, we should also pay attention to the disclosure of relevant information. On the user side, the user's cognition, attitude, and behavior of personal information risks when participating in interaction are the basic elements to be included in the interaction model to protect the user's personal privacy information. On the enterprise side, the appropriateness of its data behavior and the integrity of its protection are feasible and effective guarantees for the protection of personal privacy information. The data mining model of personal privacy protection is shown in Figure 1.

The data provider has shifted from service organizations to individuals as a result of the rapid adoption of personal smart devices, and traditional privacy protection methods are no longer adequate for the protection of personal privacy data. To achieve effective personal information protection, we must first clarify the most basic data behavior and provide the most practical reference from the enterprise behavior and regulation level. To solve the problem of personal data protection in particular, we must first address the problem [23]. The method of data encryption encrypts data while also completing complex calculations with the help of secure multi-party protocols, as the name implies. The difficult assumption of encryption algorithm and protocol construction underpins security. In academia and industry, the privacy difference is the most common method for protecting data privacy and the evaluation standard for privacy schemes. This model assumes that the adversary has sufficient background knowledge and that the addition or deletion of any record has no impact on the query's final result. Differential privacy protection technology is a well-defined privacy protection model that can withstand all attacks based on assumptions about background knowledge. Its main principle is to achieve privacy protection by adding random noise to distort the original data while maintaining the original data's statistical characteristics. Differential privacy mainly distorts data by adding noise to protect privacy. Privacy difference is independent of the background knowledge of the adversary, and it can provide a stronger privacy protection ability than the traditional anonymous protection mechanism. However, the differential privacy protection technology is difficult to be applied to the application scenarios where multiple data owners do not collude.

The server aggregates the user's personal disturbance reports from the client and decodes them to obtain valuable statistical information, while local privacy sets the privacy protection mechanism directly at the client. To avoid the privacy leakage of the untrusted third-party server, this process does not need to collect the client's real original data information, and it can be applied to a variety of complex collection scenarios. Although differential privacy protection technology improves privacy protection to some extent, noise introduces changes in the original data distribution, reducing the accuracy of results and data availability. Differential privacy technology can be used to store databases, effectively resolving the local storage privacy security problem [24]. Differential privacy, on the other hand, resolves the local storage privacy leakage problem. Secure multiparty computing is based on the assumption that multiple service users who do not trust each other exchange data information via secure multiparty protocols, allowing each service user to perform distributed machine learning tasks based on their own data. Federated learning, as a distributed machine learning framework, aims to train a high-quality centralized model while keeping local training data distributed on clients and allowing multiple users to train the same learning tasks at the same time. Each user downloads the global model, calculates the local model's update using the local data set, and uploads the update to the central server at the end of each training round. To calculate a new global model, the central server combines the local updates from clients.

### 3.2. Construction of Privacy Protection Model Based on Machine Learning

Machine learning is a branch of artificial intelligence. Machine learning is a scientific study of algorithms and statistical models used by computer systems to gradually improve the performance of specific tasks. The machine learning algorithm is a mathematical model based on the so-called “training data set.” It can complete forecasting or decision-making problems without the guidance of a specific program. Most of the traditional machine learning training algorithms are only suitable for single machine learning. Therefore, machine learning in the distributed environment needs the corresponding distributed machine learning platform to complete. Machine learning algorithms are closely related to computational statistics. Machine learning problems can often be attributed to an optimization problem. The theory of optimization provides a theory and method for machine learning. In machine learning security, the adversary model is often used to describe the strength of an adversary. Distributed machine learning has three advantages: ① using data distributed in different nodes to train the model together increases the accuracy of the model. ② Storage units distributed in different nodes are used to store data, which increases the data set capacity for model training. ③ The computing units distributed in different nodes are used for training, which enhances the computing ability of the system itself. Machine learning is widely used in data mining, computer vision, e-mail filtering, detection of credit card fraud, and medical diagnosis and analysis. While machine learning is widely used in various fields, it also brings many threats to security and privacy. Generally speaking, learning in machine learning can be divided into three categories: supervised learning, unsupervised learning, and reinforcement learning. In supervised learning, the machine learning algorithm is based on a set of data sets with standard input and output. Supervise the use of data of known labels or classes. In unsupervised learning, the algorithm establishes a mathematical model of a set of data, which only contains the input but not the expected output. Reinforcement learning is based on the maximization of some scalar reward goals, based on data and some future rewards. However, this type of learning is limited to dealing with a small number of key parameters. The general process of personal information processing is shown in Figure 2.

Vector homomorphic encryption is a homomorphic encryption scheme for vector encryption. In machine learning, there are many operations for vectors. Therefore, a vector homomorphic encryption scheme is very important for machine learning. Homomorphic encryption technology is a kind of public key encryption system, which encrypts the original data to protect the privacy of data. Homomorphic encryption has its natural advantages, which makes it one of the candidates for privacy protection solutions in the era of big data. Its main advantage is that it can make the third-party complete homomorphic operation of data without decryption. The security of a homomorphic encryption algorithm is based on the difficulty assumption of the algorithm, which can provide a good security guarantee. Homomorphic encryption can encrypt both local data and model parameters. Using homomorphic encryption to support ciphertext calculation can solve the problem of machine learning by combining multiple participants' data sets and provide a data security guarantee for machine learning in a big data environment. The algorithm framework is divided into two parts: initialization and classification. Initialization includes the following steps: data preparation and data uploading; Classification includes the following steps: query matrix generation, secure similarity calculation, and secure multiparty calculation to obtain results. The homomorphic properties of subtraction and scalar multiplication of the algorithm are shown in the following formulas:

(1) $$\begin{array}{c} \left(\left(c_{1}-\ldots -c_{n}\right)-2l_{1}Z_{1}\right)\mathrm{mod}p_{3}=s^{d}\left(r_{1}p_{2}+km_{1}+l_{1}e_{1}\right)-\ldots -\left(r_{n}p_{2}+km_{n}+l_{n}e_{n}\right)\\ -\left(2r{}^{\prime }p_{2}+2l_{1}e_{1}\right)\mathrm{mod}p_{3}\\ \overset{\Delta }{=}s^{d}\left(rp_{2}+k\left(m_{1}-\ldots -m_{n}\right)-\varepsilon p_{1}\right)\mathrm{mod}p_{3}\\ \left(N\times C_{T}\right)\mathrm{mod}p_{3}=\left(N\times s^{d}\left(rp_{2}+kT\right)\mathrm{mod}p_{3}\right)\\ \overset{\Delta }{=}s^{d}\left(rp_{2}+kNT\right)\mathrm{mod}p_{3}, \end{array}$$

where *N* is a positive integer; *Z*_1_=*Enc*_*K*_^*e*_1_^(0) is a publicly available value generated by the first data owner.

The correctness of decryption is guaranteed by the following formula:

(2) $$\begin{array}{c} x={\left|\frac{S_{c}}{w}\right|}_{q}={\left|\frac{S\left(M_{x}+e\right)}{w}\right|}_{q}={\left|x+\frac{S_{e}}{w}\right|}_{q}. \end{array}$$

To recover plaintext *x* from ciphertext *c* and key *S*, the condition |*S*_*e*_/*w*| < (1/2) needs to be satisfied. Because there is the following formula:

(3) $$\begin{array}{c} \sum_{i=1}^{m}\left|S\right|e_{i}<\frac{w}{2}. \end{array}$$

Going a step further *e* is

(4) $$\begin{array}{c} \left|e\right|<\frac{w}{2m\left|S\right|}. \end{array}$$

The following formula can be obtained:

(5) $$\begin{array}{c} S_{c}=wx+e. \end{array}$$

Before clients share local parameters, the parameters are processed by a privacy-protecting and verifiable mechanism, and the processed data is shared with the cloud server, obfuscating each client's local gradient and making it difficult for the cloud to extract any useful information from the collected gradient. Furthermore, a verifiable mechanism ensures the accuracy of transmission results, allowing for the effective detection of false results produced by malicious clouds. Due to the introduction of noise, the support vector machine algorithm scheme based on differential privacy protection alters the distribution of original data, lowering the accuracy, and usability of the results. Individual user data will never leave the device if local differential privacy is used. The proposed protocol strengthens data stream privacy protection, reduces attackers' options for destroying privacy and collects useful statistical data. The central idea of this paper is to query data sets in batches. Because the homomorphic encryption scheme supports homomorphic linear transformation operation, all query vectors can be placed in the same linear transformation matrix to achieve the purpose of the simultaneous query. In order to adapt to the distributed characteristics of the system, the system adopts the distributed selection random gradient descent method to update the model parameters. The core of the distributed random gradient descent method is the distributed and cooperative deep learning protocol.

If *pk*_*l*,*i*_=*pk*_*l*,*j*_, *sk*_*l*,*i*_=*sk*_*l*,*j*_, then *i*=*j*. At this time, the ciphertext polynomial kernel function of the data object *m*_*i*_ and the support vector *g*_*j*_ can be expressed as follows:

(6) $$\begin{array}{c} p_{j,i}=K\left(SV_{j},C_{i}\right)={\left(s_{j,i}+c\left(1\right)\right)}^{u}={\left(\sum_{z=1}^{d}\left(c_{jz}^{*}⊗c_{iz}\right)+c\left(1\right)\right)}^{u}. \end{array}$$

Evaluate all ciphertexts *c*_*ij*_(*j*=1,2,3,…, *l*_*i*_) of the *i* th data owner as follows:

(7) $$\begin{array}{c} c_{i}=Eva\left(c_{i1},\ldots ,c_{il_{i}}\right)=\sum_{j=1}^{l_{i}}Enc_{K}^{e_{i}}\left(m_{ij}\right)\underset{=}{\Delta }s^{d}\left(r_{i}p_{2}+km_{i}+l_{i}e_{i}\right)\mathrm{mod}p_{3}. \end{array}$$

Evaluating the ciphertext *c*_*i*_(*i*=1,2,3,…, *n*). for all *n* data owners is

(8) $$\begin{array}{c} c=Eva\left(c_{i},\ldots ,c_{n}\right)=\sum_{i=1}^{n}s^{d}\left(r_{i}p_{2}+km_{i}+l_{i}e_{i}\right)\underset{=}{\Delta }s^{d}\left(rp_{2}+km+\varepsilon p_{1}\right);\varepsilon \in Z. \end{array}$$

The correlation error is used as a measure of an average calculation error, while MAPE is used as a measure of frequency estimation error. The absolute value of the predicted value minus the actual value divided by the actual value is the correlation error. The following is the definition of the relevant error:

(9) $$\begin{array}{c} \text{Related error}=\left|\frac{y_{i}-x_{i}}{x_{i}}\right|\times 100\%. \end{array}$$

The absolute value of the difference between the estimated and real frequencies is known as MAPE. Divide the absolute value by the real frequency, then add these numbers together and divide by the data range's length. The following is the MAPE definition:

(10) $$\begin{array}{c} \text{MAPE}=\frac{\sum_{i=1}^{\left|D\right|}\left|\left(y_{i}-x_{i}\right)/x_{i}\right|}{\left|D\right|}\times 100\%. \end{array}$$

The ciphertext of personal data is of no use to individuals and needs to be kept confidential to other data owners. Therefore, the decryption algorithm of the ciphertext of personal data is abandoned in the design. In this paper, the algorithm classifies the test data set by calculating the similarity between the test data set and the training data set. The test data set selects the most similar *k* data from the training data set, and these *k* data confirm the label of the test data by voting mechanism. Privacy difference realizes privacy protection by adding noise to the survey results, and the added amount of noise not only protects users' privacy but also keeps data availability, so sensitivity becomes the key parameter of noise control. In local differential privacy, the concept of sensitivity is based on any two pieces of data. The mining sharing method similar to secret sharing in the algorithm is to prevent the fall and conspiracy attacks. The sharing method ensures that different data owners have different personal keys. Therefore, only when the databases of all the data owners participating in the mining are spliced into a joint database can the ciphertext mining results be decrypted correctly.

## 4. Result Analysis and Discussion

The privacy stream is released in real time using sliding window technology in this paper. It lowers computing and storage costs while also lowering privacy budget consumption when compared to traditional privacy protection methods. The proposed protocol adaptively determines the window length of the stable subdata stream, detects significant movement, opens a new window in time, and captures the trend and distribution of the data stream to further reduce storage space and better allocate the privacy budget. This section examines the antiattack performance of this scheme as well as several comparison schemes in order to verify the security of this method. The performance of these schemes against attacks is detailed in Table 1.

It can be seen that this scheme can defend against more types of attacks and has higher security. In the distributed selection random gradient descent method, a small number of local model parameters are selected to update in each iteration, and this selection process is completely random. The distributed random selection gradient descent method assumes that there are two or more participants, who are independent of each other and participate in the training in parallel. After each round of local training, participants share the gradients of the calculated parameters, and each participant completely controls which gradients to share and how often to share them. To verify the impact of privacy budget on usability in real data sets, different algorithms are used to conduct experiments on real data sets.  Figure 3 shows the impact of the privacy budget on evenly distributed data sets.  Figure 4 shows the impact of the privacy budget on real data sets.

Experiments show that under different privacy budgets, the usability of this algorithm is higher than that of the other two algorithms, which proves that this algorithm is also feasible in practical application. The data encryption stage is a constant complexity operation. After the encrypted data is processed, the future expenses mainly come from the data query users. As for secure multiparty calculation, the steps to obtain the results are clear and simple, so the efficiency is very high. In the comparative evaluation stage, this paper does not consider the two stages of data preparation and secure multiparty calculation to obtain the results. Different schemes are applied to personal information privacy protection, and their security performance is compared. The results are shown in Figure 5.

The method in this paper is safe and has some practical application value, according to the data in Figure 5. Significant movement in the data stream indicates the occurrence of a new event or trend. The newly observed tuples can be added to the current window to form a stable subdata stream if they maintain the current window's stability. A new window should be opened if new trends in the data stream emerge.  Table 2 compares the results of various algorithms in terms of performance.

It can be seen that the performance of this algorithm is generally better than other comparison algorithms. Many participants in the system participate in the training on the same combined data set to complete machine learning and ensure that no local information of the participants is leaked to the central server during this process.  Figure 6 is the simulation diagram of the secure distance calculation protocol.

From the data analysis, it can be seen that the decision-making process of the scheme classification in this paper is completely outsourced, and the data belonging to the master only needs to undertake the encryption in the initial stage and the decryption in the result acquisition stage. Comparing the adaptive framework algorithm and homomorphic encryption algorithm with the algorithm in this paper, the accuracy of different algorithms is shown in Figure 7.

It can be seen that the accuracy of this algorithm is higher than that of the adaptive frame algorithm and homomorphic encryption algorithm, and it has a certain superior performance. The experimental results show that the proposed protocol has high practicability, which is applicable to both numerical attributes and classified attributes and can keep its practicability under different distributions and data stream sizes. This algorithm has a fast convergence speed, and the average error rate decreases by 4.17% compared with the traditional algorithm. Moreover, the accuracy of this algorithm reaches 95.37%, which is about 8.76% higher than the previous algorithm. The scheme proposed in this paper has obvious advantages. At the same time, it realizes multidata ownership setting, complete outsourcing calculation, and zero communication consumption. At the same time, it supports the inner product kernel function and polynomial kernel function classification. This scheme can not only protect the privacy of the stream, but also ensure high practicability, and the overhead of storage and computing power is small.

## 5. Conclusions

In view of the threats to personal information privacy, we need to further explore the defense technologies against poisoning attacks, confrontation attacks, and other attacks, improve the robustness of the model, and study the defense means against stronger attacks. In this paper, aiming at the existing privacy protection of personal information, combined with the research status at home and abroad, the machine learning platform and homomorphic encryption scheme are studied, respectively. By observing the characteristics of big data and the new publishing mode, this paper analyzes the potential risks of privacy leakage caused by data association analysis. Then, the privacy protection criterion matching its characteristics is studied, and the user's demand for data privacy protection and data availability is understood, and a privacy protection model based on machine learning is constructed. A privacy protection mechanism based on elliptic curve and homomorphic encryption is designed to cover the local gradient of each client, which makes it difficult for malicious adversaries and semitrusted cloud to reason the original information of the data set. The proposed privacy protection mechanism keeps the high prediction accuracy of the training model and balances the security and efficiency well. In this paper, based on vector homomorphic encryption, the similarity measure of vectors under ciphertext is designed. It has the advantages of low interaction cost, safety, and high efficiency. In order to verify the performance of the algorithm, a lot of experiments are carried out. The experimental results show that this algorithm has a fast convergence speed, and the average error rate decreases by 4.17% compared with the traditional algorithm. Moreover, the accuracy of this algorithm reaches 95.37%, which is about 8.76% higher than the previous algorithm. Although this paper has achieved some research results, there are still some shortcomings and places to be improved in the research process. For example, the low efficiency of the data fusion operation of local model parameter group ciphertext will be improved in the followup work.

## Figures and Tables

**Figure 1:** Data mining model of personal privacy protection.

**Figure 2:** Flow chart of personal information processing.

**Figure 3:** The influence of privacy budget on evenly distributed data sets.

**Figure 4:** The impact of privacy budget on real data sets.

**Figure 5:** Security comparison of different schemes.

**Figure 6:** Simulation diagram of safety distance calculation protocol.

**Figure 7:** Accuracy comparison of different algorithms.

**Table 1:** Anti-attack performance of different security schemes.

Serial number	Attack type	Secure data aggregation scheme	Secure data mining scheme on vertically partitioned database	Mining scheme on horizontal partitioned database	The security data mining scheme in this paper
1	Ciphertext-only attack	Can defend	Can defend	Can defend	Can defend
2	Known plaintext attack	Can defend	Unprotectable	Unprotectable	Can defend
3	Select plaintext attack	Can defend	Unprotectable	Unprotectable	Can defend
4	Selected ciphertext attack	Unprotectable	Unprotectable	Unprotectable	Unprotectable
5	Unauthorized mining attack	Can defend	Unprotectable	Unprotectable	Can defend
6	Forgiveness attack	Can defend	Unprotectable	Unprotectable	Can defend
7	Unauthorized decryption attack	Unprotectable	Unprotectable	Can defend	Can defend
8	Owner fall	Unprotectable	Unprotectable	Unprotectable	Unprotectable

**Table 2:** Performance comparison results of different algorithms.

Algorithm	Average error	Recall rate	Accuracy rate
Distributed privacy protection algorithm	0.548	0.874	0.862
Adaptive frame algorithm	0.496	0.887	0.894
Homomorphic encryption algorithm	0.217	0.926	0.918
*K*-means clustering algorithm	0.301	0.894	0.901
Algorithm in this paper	0.131	0.963	0.954

## Data Availability

The data used to support the findings of this study are included within the article.
